# Automatic Detection of Cases of COVID-19 Pneumonia from Chest X-ray Images and Deep Learning Approaches

**DOI:** 10.1155/2022/7451551

**Published:** 2022-09-06

**Authors:** Fahima Hajjej, Sarra Ayouni, Malek Hasan, Tanvir Abir

**Affiliations:** ^1^Department of Information Systems, College of Computer and Information Sciences, Princess Nourah bint Abdulrahman University, P.O. Box 84428, Riyadh 11671, Saudi Arabia; ^2^Ajloun National University, Ajloun, Jordan, Iraq; ^3^The University of Mashreq, Research Center, Baghdad, Iraq; ^4^Department of Business Administration, Faculty of Business and Entrepreneurship, Daffodil International University, Dhaka, Bangladesh

## Abstract

Machine learning has already been used as a resource for disease detection and health care as a complementary tool to help with various daily health challenges. The advancement of deep learning techniques and a large amount of data-enabled algorithms to outperform medical teams in certain imaging tasks, such as pneumonia detection, skin cancer classification, hemorrhage detection, and arrhythmia detection. Automated diagnostics, which are enabled by images extracted from patient examinations, allow for interesting experiments to be conducted. This research differs from the related studies that were investigated in the experiment. These works are capable of binary categorization into two categories. COVID-Net, for example, was able to identify a positive case of COVID-19 or a healthy person with 93.3% accuracy. Another example is CHeXNet, which has a 95% accuracy rate in detecting cases of pneumonia or a healthy state in a patient. Experiments revealed that the current study was more effective than the previous studies in detecting a greater number of categories and with a higher percentage of accuracy. The results obtained during the model's development were not only viable but also excellent, with an accuracy of nearly 96% when analyzing a chest X-ray with three possible diagnoses in the two experiments conducted.

## 1. Introduction

COVID-19, a new type of coronavirus, was discovered in lower airway samples from several patients in Wuhan, China, in December 2019 [1]. Fever, fatigue, a dry cough, and difficulty breathing were among the symptoms of severe pneumonia in these patients. It is believed to have originated in a seafood market in Wuhan. The spread of this virus created a situation that the World Health Organization classified as a pandemic (WHO). The incubation period was estimated to be 5.2 days, allowing the disease to spread globally via air travel. Evidence suggests that the virus can be transmitted during the incubation period in asymptomatic patients. [2] The virus can be spread from person to person through droplets from infected patients' noses and mouths or through contact with contaminated surfaces.

More than 6 million confirmed cases of COVID-19 have been identified worldwide as of this writing, and multiple case reports have suggested that COVID-19 can be transmitted before symptoms appear. An infectious virus has also been found in presymptomatic COVID-19 cases [3]. While the level of infectious virus required for efficient transmission is unknown, detection of infectious virus extracted from upper airway samples suggests that COVID-19 transmission can occur before symptoms appear.

Many cities, state, and federal leaders have called for more real-time reverse transcription-polymerase chain reaction tests to check for the presence of RT-PCR (Reverse Transcription Polymerase) virus genetic material in response to increased transmission. Researchers used chain reaction and serological assays to identify asymptomatic cases and potential spreaders [4].

Only people with severe disease symptoms are included in the Ministry of Health's current testing recommendations in Iraq. For the Iraqi population, the number of tests currently available is insufficient. Patients have been diagnosed after seven days, according to reports. The real-time Reverse Transcription Polymerase Chain Reaction (RT-PCR) test, which can detect SARS-CoV-2 RNA from airway samples, is the most common method for detecting COVID-19 cases. Although the RT-PCR test is highly specific, it is performed in a manual, time-consuming, laborious, and complicated process.

Furthermore, the current limitation of population-based tests in some countries, such as Iraq, emphasizes using auxiliary methods to identify COVID-19 positive cases. The X-ray examination, in which chest X-ray images (e.g., chest X-ray (CXR) or computed tomography (CT)) are taken and analyzed by radiologists to look for indicators, is another method of identifying COVID-19 [5]. SARS-CoV-2 virus infection causes visual symptoms. Patients with abnormalities on chest radiographs, typical of people infected with COVID-19, were found in early studies, suggesting that radiographic examination could be used as a primary tool for screening for COVID-19 in epidemic areas [6]. However, detecting pneumonia on chest radiographs is a difficult task for humans to complete; it is dependent on the availability of specialized radiologists, and it is done manually and takes time. The motivation for the work in question arises at this point, which aims to present a model for automatically detecting pneumonia due to COVID-19 from chest X-rays, which is a simple task for the model, which can detect with a high percentage of precision. It is a tool that can be used in conjunction with more conclusive tests as a supplement. Machine learning [7] is already being used as a resource for disease detection and health care as a supplement to help with a variety of problems that arise in daily life. The advancement of deep learning techniques and a large amount of data available enabled algorithms to outperform medical teams in certain imaging tasks, such as pneumonia detection, skin cancer classification, hemorrhage detection, and arrhythmia detection. The main concepts discussed in this work will be presented. Initially, the possibility of identifying cases of COVID-19 using X-ray images of the chest of patients will be described. Next, we talk about machine learning, deep learning, and convolutional neural networks, which are the basis of the study of the present work. Finally, the topic related to the VGG-19 architecture is addressed, which has its main applicability in the context of pattern recognition in images having a pretrained model.

### 1.1. Identification of COVID-19 from Radiography Images

The majority of medical associations do not support the use of imaging modalities to screen patients with clinical suspicion of COVID-19. Computed tomography of the chest (CT) is recommended only for symptomatic hospitalised patients and portable chest radiography in particular instances, such as inpatients who need imaging follow-up [8]. A normal chest CT scan does not rule out COVID-19, and neither does an abnormal exam confirm a clinical suspicion. An inexpensive, easy, and practical test for patients with suspected COVID-19 is a chest radiograph. Patients who are immobile or in specific conditions such as field hospitals can benefit from the method's portability, which can be used to monitor illness progression, evaluate tracheal tubes and drug infusion lines, and rule out problems like pneumothorax. Despite its availability and ease of performance, chest radiography (Figure 1) has low sensitivity in the evaluation of patients with clinical suspicion of COVID-19, ranging from 30 to 69%, with many tests being normal in mild forms of the disease. In altered exams, the main imaging findings are consolidations and low-density opacities, usually with peripheral basal predominance. Other findings, such as pleural effusion, are uncommon, and this finding was described in only 3% of patients in a study carried out by Wong et al. [9]. The peak of findings is seen around 10 to 12 days after the onset of symptoms, and the pulmonary changes may be of rapid progression, with the evolution to the middle and upper fields or diffuse pulmonary involvement, similar to that found in the diffuse alveolar damage of the syndrome of acute respiratory distress.

Patients with respiratory problems frequently have X-ray scans of their chests taken as part of their usual care. Because of the advantages listed above, portable chest radiography will become increasingly important as COVID-19 progresses.

### 1.2. Machine Learning

Computers can learn without being explicitly programmed thanks to machine learning, which is a topic of research. Algorithmic induction is a step in the process of discovering new knowledge, and it is frequently referred to as “machine learning” when discussing this endeavour [10].

Induction is the process of creating a general model from a set of data. Induction can be associated with deduction; however, induction assumes a collection of facts and creates a general rule or model. Inductive learning is performed by reasoning about examples provided by a process external to the learning system.

The inductive learning process can be divided into the supervised learning process and the unsupervised learning process. In the supervised learning process, the inductor is provided with a set of training examples for which the associated class label is known. In general, the structure of each example is composed of a vector of characteristic values and the associated class label. The idea is to use this information in the induction algorithm to build a classifier that has the ability to identify the class of new unlabelled examples correctly. In the unsupervised learning process, the work works as follows: The inducer tries to determine if some of them can be grouped somehow from the given examples. After building these groups, an analysis is usually required to identify the context of each group within the situation being addressed.

Machine learning is at a very early stage in the process of discovering new information. Induction algorithms and other algorithms with the capacity to learn are the focus of machine learning, a scientific topic. In artificial intelligence, machine learning is a development in pattern recognition and computer learning theory. Human-like jobs can now be performed by machines, thanks to this research. But it is built on a foundation of previously learned principles that allow computers to make decisions based on a large amount of data.

### 1.3. Deep Learning

In machine learning, models are trained to perform useful tasks based on manually refined features from raw data. That is, it is necessary that the features used go through a feature engineering process so that it is possible to perform the classification or use features that were previously learned by another model. In deep learning, computers have the ability to identify useful features for the model automatically, directly from the raw data, bypassing the difficult step of manual information refinement. The main feature of the deep learning method is the focus on automatically learning data representations. This is the main difference between deep learning and traditional machine learning approaches. Resource discovery and task execution are merged into an issue and enhanced during the same training process [11].

### 1.4. Convolutional Neural Networks (CNNs)

Deep learning has sparked attention as a result of the study and application of convolutional neural networks in medical imaging. The Convolutional Neural Network is a type of artificial neural network that preserves spatial correlations in data by having fewer connections across layers [12]. The convolutional network's layers keep track of the data's relationships as it is fed in. The architecture utilised in the technique without transfer of learning is more advanced than Duran-Lopez et al. model, but less advanced than Ozturk et al. model. The model utilised was proposed in Toni work and was chosen because it is a middle architecture between the two works, allowing for a better balance between overfitting and underfitting. Each layer operation operates on a small region of the previous layer as shown in Figure 2, the flow of a traditional convolutional network. These networks enable highly efficient input data and are very effective in image-oriented tasks. In the architecture of a CNN, several layers of activation and conversion operations are interleaved. Its training process is done using backpropagation and gradient descent.

### 1.5. VGG-19

The VGG architecture was proposed based on the AlexNet architecture–the architecture with the best performance in ILSVRC 2012 and has become a milestone in the use of Convolutional Neural Networks [13]. The main feature covered in is depth. It is shown that a greater number of features can be extracted using architectures with more layers of convolutions and small convolutions (3 × 3, in this case). As a result, the VGG-16 architecture–16-layer VGG with synaptic weights–achieved great results at the 2014 ILSVRC, and although it did not win the competition, it has become one of the most used architectures in recent years, both VGG-16 and VGG-16, VGG-19. This architecture receives an RGB image of dimensions 224 × 224. ImageNet's 1.2 million general images with more than 1,000 different categories were merged into the dataset to train the VGG-19 model's 143 million parameters. The VGG-19 has a total of 19 layers for training, including convolutional and fully connected ones. The CNN VGG-19 architecture is shown in Figure 3.

## 2. Materials and Methods

This section presents the dataset chosen for the COVID-19 identification task and the proposed methodology. The model's training used chest X-ray images of patients with COVID-19, bacterial, and healthy pneumonia obtained from two distinct datasets available in the Kaggle repository: ‘Chest X-ray Images (Pneumonia)' and ‘COVID-19 chest X-ray'. The dataset was grouped into three categories: “COVID-19”, “Bacterial”, and “Healthy”. In addition to identifying COVID-19, the model proposes to identify the presence of bacterial pneumonia. The method used proposes the use of the VGG-19 convolutional neural network, which uses as a basis for training the dataset created containing the three categories described above. One of the main objectives of the work is to identify a neural network architecture capable of identifying COVID-19 with a high percentage of accuracy. In addition, the work aims to fill a gap in the literature, which consists of identifying the presence of COVID-19, bacterial pneumonia, or a healthy state. During the creation of the model, two pieces of training were carried out using the dataset, but with different volumes, which will be described in this section.

### 2.1. Datasets

Two datasets were created to be used as a database set for training. The sets were created using two different chest X-ray images of patients. A given dataset *x* has images of viral pneumonia, bacterial, and healthy pneumonia, and dataset *y* have images of COVID-19. The *x* dataset, called Chest X-ray Images (Pneumonia) and the COVID-19 chest X-ray dataset, are available on Kaggle [14]. Kaggle is a community of data scientists with several datasets available for studies, such as those used in this work. Datasets created from these distinct sources have three categories labelled “Covid-19”, “Pneumonia-Bacterial”, and “normal” in each case 266 images in dataset I and 288 images in data II set. What differs from Dataset I to Dataset II is just the volume of images contained in each one. During the selection of the images, tests were carried out to verify images that would reduce the performance.

During the selection of the images, tests were carried out in order to select images with higher quality to achieve better results during training. Images that reduced the model's performance were identified. Within the Dataset available in Kaggle, there are images with noise, noise that negatively influenced the accuracy during the tests. The selection was performed to discard images that were not frontal of the patients' chest and discard images with other noises, such as images that contained watermarks and digital arrows.  Figure 4 exemplifies images that were discarded during the image selection process to compose the dataset.

### 2.2. Image Processing and Augmentation

The images that have been selected are loaded into a list in memory where they are converted to “RGB” format using the python pillow lib and resized to a new dimension of 150 × 150 pixels. The images are all labelled with their respective categories. Using a number of data augmentation techniques, the dataset was artificially extended and improved. The data augmentation strategy avoids overfitting and improves the model's capacity to generalise during training. Data augmentation is a data manipulation technique that generates new data instances without removing the essence or core of the original data. The settings used to increase the number of images are the Rotation range (20) and Zoom range (0.15) [15–20].

The rotation interval indicates the interval in which the images were randomly rotated during training, 20°. The zoom range randomly enlarges images by 15%. In the construction of this work, the treatment of image data with the *ImageDataGenerator* 3 object of Keras was used. *ImageDataGenerator* allows you to preprocess and augment the image dataset artificially in real-time during training. Only the data augmentation techniques provided by *ImageDataGenerator* were used in this work. This is very useful, especially when the dataset is very small. The rotation and zoom techniques used in this work effectively produce more data for training [20–22]. During training, all original images are transformed over the training periods with the configuration defined in the *ImageDataGenerator* creation parameters. In each epoch, the number of images is the same as that originally entered in the training dataset, but it undergoes real-time transformations during the training. When executing this procedure, new data are created artificially for training.

All experiments performed in this work were trained using 100 epochs as a parameter. It is possible to say that 100 different versions of each original image were used during the training. The created images are not completely different from the original ones, but they have a wide variety of modifications when rotated and zoomed in on. Because it is trained on a variety of versions of the same image, the resulting model will be more robust and accurate.

### 2.3. Segregation of Images

The segregation of images for training and testing is performed randomly, where 80% of the total dataset of chest X-ray images is destined for training the model, and the remaining 20% is used for its testing.

### 2.4. Neural Network Architecture

The model was created to identify the proposed problem having VGG-19 as a base, which is a convolutional neural network architecture with very small convolution filters (3 × 3) and with 19 layers in the base model, with the weights calibrated by the image net configuration.

#### 2.4.1. Callback Functions

The ReduceLROnPlateau function was added to the model, which is a callback function that helps to reduce the learning rate by the factor, if there is no change in the loss. The configuration made for this function was to monitor the accuracy value given a configurable time *X*. In the experiment performed, this configured time was 2. If this time is reached without changing the accuracy value, the ReduceLROnPlateau will be applied given the configured factory. In the experiment, the factor configured for the function was 0.3.

#### 2.4.2. Hyperparameters

During training, hyperparameters can be used to customise many components of the learning algorithm, which can have an impact on the final model's performance and accuracy. The hyperparameters used in the model tested in this work are batch size (34); Input Shape (150 × 150 × 3); Random State (42), and 100 epochs. The Batch size parameter configures the number of images per batch in processing. The value of the input shape parameter is used to configure the input shape. Given the configured value, the random state parameter is used to reproduce the experiment. Alpha is the parameter that determines the learning rate and finally, the Epoch parameter configures the number of times the model will be trained.

#### 2.4.3. Model Layers

This section describes the actual construction of the model, detailing the layers that were added. First, the sequential model was created by adding the VGG-19 model as a base.

The pooling configured for the model was made from a resolution by the global average of two dimensions. Adding batch normalization to the process increases the stability of the neural network by applying normalizations in the middle of training. The Flatten configuration was another layer added to the configuration, which serializes the image to the dense layer. A dense layer was also added to the construction of the model, adding 64 neurons with RELU activation. A dropout with a value of 0.4 was used in the configuration of the model; the dropout serves to improve the generality of the network. The last layer added was a dense layer with 3 neurons with softmax activation [23, 24].

#### 2.4.4. Model Compilation

The parameters used when compiling the model are shown in Table 1.

Adam optimization is an optimization configuration for stochastic gradient descent based on the adaptive estimation of first- and second-order moments. The purpose of loss functions is to calculate the amount that a model should seek to minimize during training; the parameter setting chosen was binary cross-entropy which calculates the cross-entropy loss between true labels and predicted labels. The metric is a function used to judge the performance of your model and in this case, it is based on the accuracy (“acc”) of the model that measures the frequency of predictions that match the labels.

## 3. Experiments and Evaluation of Results

In this section, the experiments performed are described and their results analyzed. The first experiment was performed using “Dataset I” with 798 images for training. The second experiment was performed using the second training dataset, “Dataset II”, with a total of 864 images. What differentiates the two experiments is only the amount of data offered for training the model. The metrics used to demonstrate the results of the two experiments were: Graph of the model's precision curve, which demonstrates the accuracy performance of the model training over the epochs; Confusion matrix, the confusion matrix demonstrates the complete classification accuracy of the model; Receiver Operation Characteristic Curve (ROC) and AUC Curve: For the classification case, the ROC curve demonstrates the model's performance in distinguishing positive and negative cases. The AUC curve is derived from the ROC curve (“area under the ROC curve”), and the result is arrived at by calculating the “area under the curve”; its value varies from 0.0 to 1.0. The higher the AUC, the better the model performance.

### 3.1. First Experiment

In the task of automatically identifying COVID-19, Bacterial Pneumonia, or a healthy case through chest X-ray images of patients, the model proposed in his first experiment used a dataset with a total of 798 images, 266 of which chest X-ray images of healthy patients, 266 images of COVID-19, and 266 images of bacterial pneumonia.

The data augmentation strategy was applied in real time and during the training, the model reached an accuracy of 0.9608. The accuracy model was also generated to demonstrate the performance during the training of the epochs Figure 5(a).

A confusion matrix was generated to demonstrate the test results Figures 6(a) and 6(b) in which the zero index means bacterial pneumonia; the index 1 means COVID-19 and the index 2 indicates a normal situation. Finally, to demonstrate the performance of the first experiment, the ROC curve metric is shown in Figures 7(a) and 7(b).

### 3.2. Second Experiment

The second experiment used a dataset with 864 images for training, 288 images of chest X-rays of healthy patients, 288 images of COVID-19, and 288 images of bacterial pneumonia. The real-time data augmentation strategy was applied. During training, the model reached an accuracy of 0.9686. The accuracy model was generated to demonstrate the performance during the training of the epochs Figure 5(b). To demonstrate the test results, a confusion matrix was generated.

(Figure 5) where index zero means bacterial pneumonia, index 1 means COVID-19 and 2 normal. Finally, to demonstrate the performance of the second experiment, the curve metric ROC Analysis of results is shown in Figure 7. In the task of automatically identifying COVID-19, Bacterial Pneumonia or a healthy case through X-ray images, a model was built with the configuration described in this work. The model can be subjected to training using datasets with different volumes as a data source. This was the focus assessed in the current study experiment.

The model was subjected to training using two datasets with different volumes. Dataset I was used with a lower volume than Dataset II to identify the model's ability to improve its accuracy when subjected to training with larger datasets.

The first experiment using Dataset I generated an accuracy result of 0.9608, in the second experiment using Dataset II presented an accuracy result of 0.9686. These results were created to provide a better view of the comparison of results between experiments.

## 4. Conclusions

Intending to develop alternatives for the diagnosis of COVID-19, which has proved to be a public health problem worldwide, and seeking approaches that made this diagnosis possible with the use of deep learning, the present work analyzed several articles as a way of evaluating the feasibility of developing the proposed project. After a thorough analysis, it is possible to state that the imaging diagnosis of cases of severe acute respiratory syndrome based on X-ray exams is possible and has the possibility of differentiating it from bacterial pneumonia.

The results obtained during the development of the model proved to be viable and presented excellent results, with an accuracy of approximately 96% when analyzing chest X-rays with three possible diagnoses in the two experiments performed.

This work acts differently from the related works that were studied during the developed experiment. These works can perform a binary classification between two categories. An example is COVID-Net, which was able to identify a positive or healthy case of COVID-19 with an accuracy of 93.3%. Another example is CHeXNet, which can identify cases of pneumonia or a healthy situation in a patient with an accuracy of 95%. The current study, through experiments, proved to be efficient in detecting a greater variety of categories and with an even higher percentage of precision than the works cited. In future work, the objective is to carry out more experiments, more extensively validate the model developed and investigate the possibility of identifying other types of viral pneumonia to extend the diagnostic capacity of the model.

It will also be interesting to look for a dataset with a larger volume for training since the disease is recent, but a remarkable dataset is already available. However, with time, the tendency is to have more and more data to work within studies. Other artificial neural network architectures will also be implemented to evaluate possibilities for improvements, or even the development of a control system, to enable a safer diagnosis.

## Figures and Tables

**Figure 1:** Example chest X-ray image of: (a) Healthy. (b) Bacteremia. (c) Viral pneumonia. (d) COVID-19 viral infection.

**Figure 2:** Building blocks of a traditional CNN.

**Figure 3:** Example of the VGG-19 model network architecture.

**Figure 4:** Example of images discarded in the selection process because they contain noise.

**Figure 5:** Model Accuracy. (a) First experiment. (b) Second experiment.

**Figure 6:** Confusion matrix. (a) First experiment. (b) Second experiment.

**Figure 7:** Receiver Operation Characteristic Curve (ROC). (a) First experiment. (b) Second experiment. (Class 0 = Bacteremia group; Class 1 = COVID-19 group and Class 2 = Healthy group).

**Table 1:** Compilation parameters.

Parameter	Configuration
Adam	Optimizer
Loss	Binary cross-entropy
Metrics	acc

## Data Availability

The data used to support the findings of this study are included within the article.
